RETRACTED

# Bioinformatic Characterization of Whole Blood Neutrophils in Pelvic Inflammatory Disease: A Potential Prognostic Indicator for Transumbilical Single-Port Laparoscopic Pelvic Abscess Surgery

**DOI:** 10.1155/2022/2555603

**Published:** 2022-04-01

**Authors:** Haining Li, Yanling Hu, Dan Liu, Juanjuan Wang, Panpan Han, Nan Zhang, Yan Li

**Affiliations:** ^1^General Hospital of Ningxia Medical University, China; ^2^Ningxia Medical University, China

## Abstract

The purpose of this research is to determine the prognosis of patients treated with transumbilical single-port laparoscopic surgery for acute pelvic inflammatory illness. Postoperative data on 129 patients treated with laparoscopic surgery for acute pelvic inflammatory illness were obtained retrospectively. It was observed that the shorter the time required for postoperative leukocyte recovery to normal, the shorter the time required for postoperative pain and diet recovery, as well as hospital stay, in such individuals. CIBERSORT was used to examine patient data from GEO. The most significant difference between the normal and pelvic inflammatory groups was in neutrophil content. Association study found a substantial positive correlation between the quantity of neutrophils infiltrating the immune system and the abundance of monocyte M0 infiltrating the immune system. Neutrophil immune infiltration was strongly inversely linked with plasma cells, activated CD8+ Tm cells, and active CD4+ Tm cells. Four mRNAs linked with pelvic inflammatory illness were revealed to be strongly associated with neutrophil immune infiltration, notably *CALML4*, *COQ10B*, *DCPS*, and *PPP2R1A*. The ROC revealed that *CALML4* (area under the curve (AUC): 0.769, 95% confidence interval (CI): 0.638–0.881), *COQ10B* (AUC: 0.742, 95% CI: 0.587–0.881), *PPP2R1A* (AUC: 0.733 95% CI: 0.593–0.857), and *DCPS* (AUC: 0.745, 95% CI: 0.571–0.900) were potential markers for predicting pelvic inflammatory disease. *CALML4*, *COQ10B*, *PPP2R1A*, and *DCPS* may be critical determinants determining the amount of preoperative neutrophil infiltration and the time required for leukocyte recovery after single-port laparoscopy in acute pelvic inflammatory illness.

## 1. Introduction

The acute pelvic inflammatory disease involves an acute inflammatory lesion in the female internal genitalia and surrounding connective tissue, which is caused by the invasion of pathogenic bacteria, viruses, mycoplasma, and chlamydia [1, 2]. The principal clinical manifestations of acute pelvic inflammatory disease are lower abdominal pain, fever, and increased vaginal discharge [3]. It occurs rapidly and is characterized by several symptoms, including acute endometritis, acute pelvic peritonitis, and acute tubal inflammation [4–7]. Acute pelvic inflammatory disease can easily persist and evolve into chronic pelvic inflammatory disease if not treated thoroughly, even leading to permanent sequelae such as tubal infertility and ectopic pregnancy [8]. Moreover, acute pelvic inflammatory disease can develop into diffuse peritonitis, pelvic abscess, septicemia, and infectious shock if not treated promptly, which can be life-threatening in severe cases [9].

RETRACTED

Laparotomy and laparoscopic surgery are effective means of treating pelvic abscesses. Compared with laparotomy, laparoscopic surgery is characterized by less bleeding, higher safety, faster recovery, shorter hospital stay, lower rate of postoperative wound infection, the lower recurrence rate of chronic pelvic pain, and pelvic inflammatory disease [10]. Compared with the traditional multiport laparoscopic technique, the single-port transumbilical laparoscopic technique has the advantage of smaller incisions, less damage, and less postoperative pain [11, 12]. The efficacy of the transumbilical single-port laparoscopic technique in treating pelvic abscesses and its long-term functional recovery still needs to be studied in more detail for reaching a consensus. Indicators that can effectively reflect the prognosis of surgical outcomes should be identified.

The leukocyte count is one of the most important clinical indicators of the inflammatory status of the body and can be used as an indicator of pelvic inflammatory disease [13, 14]. In clinical practice, we have observed that postoperative leukocyte recovery time reflects the surgical efficacy of transumbilical single-port laparoscopy for pelvic abscesses. Leukocyte bioinformatic profiling is an important method for finding biomarkers of efficacy after single-port laparoscopic treatment of pelvic abscesses. It was found that cellular immunity played a dominant role in the infection process, and the levels of IL-2 were significantly increased in the blood of rats with pelvic inflammatory disease [15]. Therefore, immunoinfiltration analysis is an effective method for determining the prognosis of acute pelvic inflammatory illness. Bioinformatics is a new discipline formed by combining life sciences and computer science [16]. Bioinformatic analysis has been successfully used to identify important biomarkers for various diseases [17, 18].

To effectively assess the efficacy of transumbilical single-port laparoscopic pelvic abscess surgery, we proposed combining clinical and bioinformatic data to perform bioinformatic characterization of whole blood leukocytes and to identify biomarkers potentially associated with the prognosis of acute pelvic inflammatory disease.

RETRACTED

## 2. Materials and Methods

### 2.1. General Information

In this study, we retrospectively analyzed patients from the General Hospital of Ningxia Medical University who were treated with laparoscopic surgery for acute pelvic inflammatory disease from January 2019 to June 2021. The inclusion criteria were as follows: (1) patients who met the diagnostic criteria for acute pelvic inflammatory disease [19], (2) those who had abdominal pain or pelvic mass, (3) those who signed informed consent for the study, and (4) those who were treated with transumbilical single-port laparoscopic pelvic abscess surgery. The exclusion criteria were as follows: (1) patients who had serious organ insufficiency, (2) those who had gynecological malignancies, (3) those who had psychiatric disorders and cognitive impairment, and (4) those who refused to participate in this study. The surgeries were performed by Yan Li, the corresponding author of this study. The study included 129 patients. The study was approved by the Ethics Committee of the General Hospital of Ningxia Medical University. Informed consent was obtained from the patients and their families. Leukocyte recovery time is the time it takes for the postoperative leukocyte count to recover from abnormal to 4.0‐10.0 × 10^9^/L and the neutrophil ratio to return to normal.

### 2.2. Data Acquisition

The dataset was obtained from NCBI's Gene Expression Omnibus (GEO) database. GEO is a public repository of functional genomics data and provides tools to help users query and download experimental and curated gene expression profiles. The datasets were selected based on the following eligibility criteria: (1) containing at least 10 samples, (2) containing at least 5 cases and 5 controls, and (3) providing raw data or arrays of datasets. GSE110106 is a dataset for studying the transcriptomic specificity of blood from patients with pelvic inflammatory disease [20]. Data from 47 normal and 7 non-STI cases of pelvic inflammatory disease in GSE110106 were extracted for analysis.

### 2.3. Screening for Differentially Expressed Genes (DEGs)

To eliminate heterogeneity across platforms, the raw gene expression data downloaded from the GEO database were first preprocessed, and all data were normalized. After determining that the data could be compared using principal component analysis (PCA), they were uploaded to the website iDEP.91 (http://bioinformatics.sdstate.edu/idep/) in order to screen for differences in whole blood gene expression between healthy individuals and patients with pelvic inflammatory disease. After uploading the collected data, the species “Human” was chosen and the data type “Normalized expression values” was chosen. Additionally, DEGs were screened. *p* values less than 0.05 were deemed significant.

RETRACTED

### 2.4. Immunoinfiltration Analysis

A leukocyte gene signature matrix (LM22) was downloaded from CIBERSORT (http://cibersort.stanford.edu/) as in previous researches [21–25]. The CIBERSORT method was used to determine the percentage of 22 immune cell infiltrates in each patient's blood sample with pelvic inflammatory illness. To display and analyze the degree of immunological infiltration, the R software packages “BiocManager” and “vioplot” were utilised.

### 2.5. Enrichment Analysis

To understand the function of the target gene cluster and the pathogenesis of the disease, GO functional annotation and KEGG pathway enrichment analysis were performed on the screened DEGs [26]. GO divides the function of a gene into 3 components: cellular component (CC), molecular function (MF), and biological process (BP). KEGG is an online database for understanding higher-level functions and biological systems (e.g., cells, organisms, and ecosystems) and screening for signaling pathways that are significantly associated with DEGs. The R software ggplot2 package was used for visualization.

The Kyoto Encyclopedia of Genes and Genomes (KEGG) gene set was obtained from the Broad Institute website (http://software.broadinstitute.org/gsea/index.jsp) [27, 28]. Analysis of pathway enrichment in the blood of patients with the pelvic inflammatory disease was performed using GSEA software (version 4.0.2) as in previous researches. FDR *q* value < 0.05 and *p* < 0.05 were considered significant.

### 2.6. Statistical Methods

Statistical analysis and visualization of the data were performed using R software. The “ggstatsplot” package (https://github.com/IndrajeetPatil/ggstatsplot) was used for the Spearman correlation analysis of diagnostic markers and infiltrating immune cells. The “ggplot2” and “circlize” packages (version 0.4.12) were used to visualize the results [29]. PCA was performed using R software. The key mRNAs associated with the pelvic inflammatory disease were analyzed using a support vector machine based on the R software packages “caret,” “kernlab,” and “e1071.” The seed was set to 124, and the method was “svmRadial” [30]. The *t*-test or ANOVA was used to determine the differences between the groups. The Wilcoxon test was used to determine the differences between immunoinfiltrated groups. *p* < 0.05 was judged to be statistically significant.

## 3. Results

### 3.1. Leukocyte Recovery Time Corresponds to Numerous Clinical Markers after Single-Port Laparoscopy for Acute Pelvic Inflammatory Disease

We studied the postoperative data of 126 individuals who had laparoscopic surgery for acute pelvic inflammatory illness in this research. Postoperative leukocyte recovery time was shown to be linked to postoperative pain, postoperative dietary recovery time, hospital stay duration, and hospital expense (*p* < 0.05; Figure 1). The shorter the leukocyte recovery time, the shorter the postoperative pain recovery time, postoperative dietary recovery time, and hospital stay, which also means less hospital expenditure. This suggested that leukocyte recovery time is a potential prognostic indicator for early recovery after single-port laparoscopy for acute pelvic inflammatory disease.

RETRACTED

### 3.2. Analysis of Blood Immune Infiltration in Patients with and without Pelvic Inflammatory Disease

The CIBERSORT calculation was used to analyze the proportion of 22 immune cell infiltrates in the blood sample of each patient with pelvic inflammatory disease. The dataset for this study included 54 samples, of which only 7 were non-STI pelvic inflammatory samples. The limitations of the samples could have led to no significant differences in the abundance of blood immune infiltration between patients with pelvic inflammatory disease and healthy individuals (Figure 2(a)). Further, PCA revealed no significant difference in the abundance of blood immune infiltrates between patients with pelvic inflammatory disease and healthy individuals. Neutrophils are major components of leukocytes. Correlation analysis suggested that the abundance of immune infiltration of neutrophils was significantly positively correlated with that of monocyte M0. The abundance of immune infiltration of neutrophils was significantly negatively correlated with that of plasma, activated CD8^+^ Tm, and activated CD4^+^ Tm cells (Figure 2(b)). The PCA approach was used to perform cluster analysis on these samples (Figure 2(c)). Therefore, we concluded that the difference in the abundance of blood immune infiltrates between patients with pelvic inflammatory disease and healthy individuals is mainly reflected in the difference in the degree of infiltration of neutrophils.

### 3.3. Differential Transcriptional Profiles Identified in the Blood of Patients with Pelvic Inflammatory Disease

To remove batch effects, we first preprocessed the raw gene expression data downloaded from the GEO database, and all data were normalized. PCA was used to determine that the disease and health groups were comparable (Figures 3(a) and 3(b)). Differentially expressed mRNAs (DEGs) in the pelvic inflammatory group versus the healthy group were identified and presented in a heat map (Figure 3(c)). These mRNAs included those of genes *BCLAF1*, *GLYR1*, *RNF20*, *KLF2*, *RHOA*, *PPCS*, *TBC1D23*, *LRRC20*, *KIAA1429*, *CALML4*, *DTX3L*, *PPID*, *GSDMA*, *KLLN*, *OTUB1*, *PACS1*, *PPP2R1A*, *FLNA, LSM12*, *TOR3A*, *DCPS*, *SCAND1*, *TBX21*, *CERKL*, *HEATR1*, *PRAF2*, *WTAP*, *TMEM69*, *TNRC6B*, *CCDC47*, *COQ10B*, *DERPC*, *HERPC*, *HNRNPA3*, *AAMP*, *CCDC71*, *ATF6B*, *TAF15*, *APP*, *SLC39A1*, *LYRM2*, and *RPS6KA3*. GSEA suggested that the mRNAs in patients with the pelvic inflammatory disease were significantly enriched in the KEGG TGF-beta signaling pathway, KEGG oxidative phosphorylation, KEGG leukocyte transendothelial migration, and KEGG cytokine receptor interaction (Figure 3(d)).

RETRACTED

### 3.4. Analysis of Key mRNAs Associated with Pelvic Inflammatory Disease and Immune Cell Infiltration

SVM multiple iterations suggested the highest prediction accuracy when 34 predictors are selected (Figure 4(a)). Key mRNAs associated with pelvic inflammatory disease (including those of *CALML4*, *COQ10B*, *DCPS*, and *PPP2R1A*) were found to be significantly associated with immune infiltration of neutrophils (Figures 4(b)–4(e)). *CALML4* and *COQ10B* were found to be significantly positively correlated with abundant infiltration of neutrophils, whereas *PPP2R1A* and *DCPS* were found to be significantly negatively correlated with neutrophil enrichment (Figures 4(b)–4(e) and 5(a)). Interestingly, the expression of *CALML4*, *COQ10B*, *PPP2R1A*, and *CALML4* was positively correlated with each other (Figure 5(b)). The receiver operating characteristic (ROC) curves suggested that *CALML4* (area under the curve (AUC): 0.769, 95% confidence interval (CI): 0.638–0.881), *COQ10B* (AUC: 0.742, 95% CI: 0.587–0.881), *PPP2R1A* (AUC: 0.733 95% CI: 0.593–0.857), and *CALML4* (AUC: 0.745, 95% CI: 0.571–0.900) were potential biomarkers for predicting the prognosis of pelvic inflammatory disease (Figures 5(c)–5(f)). Enrichment analysis of key mRNAs (*CALML4*, *COQ10B*, *PPP2R1A*, and *CALML4*) associated with pelvic inflammatory disease was also performed (Figures 6(a) and 6(b)). In conclusion, we identified four potential neutrophil-related biomarkers of pelvic inflammatory disease. These four biomarkers may be the key factors influencing the abundance of preoperative neutrophil infiltration in pelvic inflammatory disease and time to leukocyte recovery after single-port laparoscopy for acute pelvic inflammatory disease.

## 4. Discussion

Prognostic indicators are lacking for transumbilical single-port laparoscopic pelvic abscess surgery. In this study, we combined clinical and bioinformatic data to perform bioinformatic characterization of whole blood leukocytes and identified potential neutrophil-related biomarkers in acute pelvic inflammatory disease, which were *CALML4*, *COQ10B*, *PPP2R1A*, and *CALML4*. These four biomarkers may be the correlated factors influencing the abundance of preoperative neutrophil infiltration in pelvic inflammatory disease and time to leukocyte recovery after single-port laparoscopy for acute pelvic inflammatory disease.

RETRACTED

Neutrophils, as polymorphonuclear leukocytes, are major players in natural immunity and form an important line of defense against foreign pathogens. Neutrophils are the first cells to be recruited at the site of inflammation [31, 32]. When pathogens attack, neutrophils rapidly migrate to the site of inflammation under the action of chemokines and adhere to endothelial cells to play a phagocytic role, preventing the spread of pathogens and development of systemic inflammation [33]. Foo et al. found that neutrophils could be significant predictors of mortality in bacterial liver abscesses in a comparative study of prognosis using neutrophils and lymphocytes [34]. In this study, we found that the shorter the postoperative leukocyte recovery time, the shorter the postoperative pain recovery time, postoperative dietary recovery time, and hospital stay in patients treated with laparoscopic surgery for acute pelvic inflammatory disease, which also meant less hospital expenditure. This suggested that leukocyte recovery time is a potential predictor of recovery time after single-port laparoscopy for acute pelvic inflammatory disease. We used the CIBERSORT calculation to analyze the proportion of 22 immune cell infiltrates in the blood of pelvic inflammatory disease samples in the GEO database GSE110106 dataset and found no significant difference in abundance of blood immune infiltration between patients with pelvic inflammatory disease and healthy individuals. This could be because the dataset for this study included 54 samples, of which only 7 were non-STI pelvic inflammatory samples. Correlation analysis suggested that the abundance of immune infiltration of neutrophils was significantly positively correlated with that of monocyte M0. The abundance of immune infiltration of neutrophils was significantly negatively correlated with that of plasma, activated CD8^+^ Tm, and activated CD4^+^ Tm cells. Thus, we suggested that the difference in the abundance of blood immune infiltrates between patients with pelvic inflammatory disease and healthy individuals was mainly reflected in the difference in the degree of infiltration of neutrophils.

CALML4 is a member of the calmodulin superfamily of small EF-hand proteins. The signature “EF-hand” shape of members of the calmodulin superfamily allows them to act as calcium sensors and buffers within cells [35, 36]. *CALML4* shares at least 45% sequence identity with conventional calmodulin. A prominent function of conventional calmodulin is to act as a light chain member of the myosin family [37]. CALML4 also has been shown to associate with MYO7B [38]. Yang et al. reported that *CALML4* could be used as a prognostic biomarker for gastric cancer and patients with overexpression of CALML4 had a better prognosis than those with low expression. In *Helicobacter pylori*-positive gastric cancer, both hsa-miR-223 and hsa-miR-411 can regulate CALML4 and thus activate the CGMP-PKG signaling pathway [39]. To the best of our knowledge, this is the first study to report that *CALML4* was associated with pelvic inflammatory disease and was significantly positively correlated with the enrichment of neutrophils. The main difference in the abundance of blood immune infiltration between patients with pelvic inflammatory disease and healthy individuals was in terms of the degree of infiltration of neutrophils. The ROC curve showed an AUC of 0.769 for *CALML4* to predict pelvic inflammatory disease, suggesting that *CALML4* is a potential biomarker for pelvic inflammatory disease.

RETRACTED

COQ10B was found in the mitochondria of most eukaryotes. *COQ10* encodes a protein that affects the function of the respiratory chain by participating in transport to the mitochondria. Additionally, it is an important antioxidant [40, 41]. COQ10B has been reported to provide a degree of protection against organ damage caused by sepsis [42, 43]. Furthermore, COQ10B's antioxidant properties make it a possible treatment tool for illnesses involving the mitochondrial respiratory chain [44]. Studies have confirmed that oxidative stress injury is involved in the development of pelvic inflammatory disease, leading to cellular and tissue damage [4, 45]. The ROC curve in this study showed that the AUC of *COQ10B* was 0.742, suggesting that *COQ10B* is a potential biomarker of predicting pelvic inflammatory disease. To the best of our knowledge, this is the first study to report that *COQ10B*, a key mRNA associated with pelvic inflammatory disease, was positively correlated with the enrichment of neutrophils. Further studies are warranted to investigate the exact mechanism of interaction between *COQ10B* as an antioxidant and neutrophils involved in the inflammatory response.

PPP2R1A, a structural subunit of the protein phosphatase PP2A, is a positive regulatory protein essential for cell growth and proliferation. It plays a scaffolding and linkage role in the catalytic process of the PP2A holoenzyme [46–48]. PP2A is involved in regulating almost all physiological and pathological processes, such as cellular material metabolism, cell division, cell transformation, and apoptosis [46]. Haesen et al. and Cunningham et al. detected different mutants of *PPP2R1A* in lung cancer, breast cancer, and malignant melanoma with inhibitory effects on tumorigenesis and metastasis [49, 50]. Neutrophils are found in the tumor microenvironment of many cancers and are known as tumor-associated neutrophils (TANs) [51]. TANs were found to promote tumor invasion and angiogenesis through the release of proteases and cytokines [52, 53]. Some TANs exert a tumor growth-inhibiting effect [54, 55]. However, to the best of our knowledge, no studies are available demonstrating the interaction between PPP2R1A and neutrophils. To the best of our knowledge, we reported for the first time that *PPP2R1A* was significantly negatively correlated with the enrichment of neutrophils; this may be a correlated factor affecting the abundance of preoperative neutrophil infiltration in pelvic inflammatory disease. The ROC curve showed that the AUC of *PPP2R1A* for the pelvic inflammatory disease was 0.733, suggesting that *PPP2R1A* is a potential biomarker for pelvic inflammatory disease.

RETRACTED

Scavenger decapping enzyme (DCPS) is a nucleotide hydrolase belonging to the histidine triad (HIT) superfamily. DCPS is the first HIT family member with a clear biological function [56]. DCPS acts as a regulator of cap-dependent processes that influence mRNA metabolism, including splicing of mRNA precursors, nuclear export, translation, and mRNA degradation [57]. DCPS regulates gene expression by hydrolyzing mRNA 5′ residual cap structures and regulating the activity of other cap-binding proteins. Thereby, it protects cells from the potentially toxic effects of the accumulation of aberrant cap mRNA fragments [58, 59]. Previous studies suggested that DCPS is involved in key cellular processes in human neurodevelopment and organismal homeostasis [60]. To the best of our knowledge, a significant negative correlation between *DCPS* and enrichment of neutrophils was reported for the first time in this study. The ROC curve showed that the AUC of *DCPS* for the pelvic inflammatory disease was 0.745, suggesting that *DCPS* is a potential biomarker for pelvic inflammatory disease. Interestingly, although the correlations between *CALML4*, *COQ10B*, *PPP2R1A*, and *DCPS* and the enrichment of neutrophils were different, the expression of these four biomarkers was positively correlated with each other. The underlying mechanisms should be further investigated.

In conclusion, we reported that leukocyte recovery time was a potential prognostic indicator for early recovery after single-port laparoscopy for acute pelvic inflammatory disease. The difference in the abundance of blood immune infiltrates between patients with pelvic inflammatory disease and healthy individuals was mainly reflected in the difference in the degree of infiltration of neutrophils. *CALML4*, *COQ10B*, *PPP2R1A*, and *DCPS* were potential neutrophil-related biomarkers for acute pelvic inflammatory disease. These four biomarkers may be the correlated factors influencing the abundance of preoperative neutrophil infiltration in pelvic inflammatory disease and the time to leukocyte recovery after single-port laparoscopy for acute pelvic inflammatory disease.

RETRACTED

This study has some limitations. First, the results of this study were based on bioinformatic methods; however, the specific underlying mechanisms of the observations need to be confirmed by further experiments. Second, this was a retrospective study, and the four biomarkers *CALML4*, *COQ10B*, *PPP2R1A*, and *DCPS* derived from bioinformatic methods were not tested in clinical samples for validation. Third, there was no significant difference in the number of blood immune infiltrates between pelvic inflammatory disease patients and healthy persons, most likely owing to the database's small sample size. Therefore, immunoinfiltration analysis may be susceptible to several inaccuracies, which must be taken into account. Last, this was a single-center study, and a multicenter study is needed.

## 5. Conclusion

*CALML4*, *COQ10B*, *PPP2R1A*, and *DCPS* may be associated with preoperative neutrophil infiltration and time of leukocyte recovery after single-port laparoscopy for acute pelvic inflammatory illness.

## Figures and Tables

**Figure 1:** Correlation analysis of various pathological features after surgery for acute pelvic inflammatory disease. Pink and blue colors indicate a positive and negative correlation, respectively. ∗ and ∗∗ indicate *p* < 0.05 and 0.001, respectively.

**Figure 2:** Analysis of blood immune infiltration in patients with and without the pelvic inflammatory disease. (a) Comparison of the abundance of blood immune infiltration in patients with pelvic inflammatory disease and healthy individuals. (b) Analysis of the correlation between different immune cell infiltrations in the blood of a population. (c) Visualization of immune cell enrichment using PCA.

**Figure 3:** Transcriptional profiling in the blood of patients with pelvic inflammatory disease. (a, b) PCA plot before (a) and after (b) batch correction. (c) Heat map of differentially expressed genes in pelvic inflammatory disease; data processed by using the *z*-score. Red and blue indicate high and low expression, respectively. (d) GSEA display map of patients with pelvic inflammatory disease in a KEGG dataset significantly enriched for pathways.

RETRACTED

**Figure 4:** Analysis of key mRNA and immune cell infiltration in pelvic inflammatory disease. (a) SVM multiple iterations yield the highest prediction accuracy when 34 predictors are selected. (b–e) The key mRNAs *CALML4*, *COQ10B*, *DCPS*, and *PPP2R1A* associated with the pelvic inflammatory disease were found to be significantly associated with immune infiltration of neutrophils (*p* < 0.05).

**Figure 5:** Correlation analysis of key mRNAs associated with pelvic inflammatory disease and neutrophils. (a) A lollipop plot for correlation analysis of key mRNAs associated with pelvic inflammatory disease and neutrophils. (b) Correlation analysis of the expression of *CALML4*, *COQ10B*, *PPP2R1A*, and *CALML4*. (c–f) ROC curves indicate the potential of *CALML4*, *COQ10B*, *PPP2R1A*, and *CALML4* to predict pelvic inflammatory disease.

**Figure 6:** Enrichment analysis of key mRNAs associated with pelvic inflammatory disease: shown as bar graphs (a) and correlation linkage plots (b).

## Data Availability

Clinical study data for this study are available on reasonable request from the corresponding author. The raw bioinformatic data were obtained from the GSE110106 dataset in the GEO database.

## Abbreviations

BP: Biological process
CC: Cellular component
*DCPS*: Scavenger decapping enzyme
GEO: Gene Expression Omnibus
GO: Gene Ontology
KEGG: Kyoto Encyclopedia of Genes and Genomes
MF: Molecular function
PCA: Principal component analysis
Tm: Memory T cell.
